# Activation of TREK1 Channel in the Anterior Cingulate Cortex Improves Neuropathic Pain in a Rat Model

This article has been retracted.

**DOI:** 10.1155/2022/1372823

**Published:** 2022-09-30

**Authors:** Yuanzhi Peng, Qingqing Zhang, Hao Cheng, Saie Shen, Xiaojian Weng

**Affiliations:** ^1^Department of Anesthesiology and SICU, Xinhua Hospital, School of Medicine, Shanghai Jiao Tong University, Shanghai 200092, China; ^2^Department of Cardiovascular Surgery, Changhai Hospital, the Navy Medical University, Shanghai 200433, China

## Abstract

*Objective*. To explore the biological function and mechanism of TREK1 in neuropathic pain. Thirty-two healthy rats and rats with sciatic nerve chronic press-fitting model (chronic constriction injury of the sciatic nerve, CCI) were selected. Western blot, immunofluorescence staining, and patch clamp technique were performed to explore the biological functions of TREK1. The expression of TREK1 was decreased in the CCI model. The TREK1 channel current in the CCI model was decreased. After local administration of TREK1 channel activator in the anterior cingulate cortex area, the pain behavior of CCI rats and the expression of TREK1 protein were reversed. The expression of TREK1 was downregulated in the ACC area of CCI rats and the current of TREK1 was decreased, which played an important role in the regulation of neuropathic pain.

## 1. Introduction

Neuropathic pain refers to the pain that is triggered and caused by the primary injury and dysfunction of the nervous system [1]. It is characterized by progressive spontaneous pain, hyperalgesia, and hypersensitivity to pain [2]. This kind of intractable pain not only makes the patient miserable but also decreases the life quality. An increasing number of molecular targets in the pain pathways have been identified for the treatment of mental derangement rational pain [3, 4].

Peripheral nerve injury and central sensitization are considered the main pathogenesis of neuropathic pain. The anterior cingulate cortex (ACC) experiences pain in the forebrain-related brain regions, mainly in the occurrence of neuropathic pain, and plays an important role in the process of development [5]. The mechanism of ACC neurons involved in central sensitization is very complex, involving receptors, ion channels, cells, and all levels of the neural network system. Many studies have confirmed that the double hole family of potassium channels in TWIK-related potassium channel 1 (TREK1) channel is widely expressed in spinal cord dorsal horn neurons and in the central neurons of rats, which could adjust the excitability of nerve cells and the neurotransmitter release and may be associated with the pathogenesis of chronic pain [6, 7].

TREK1 channel could be regulated by pain stimulation, including pressure, and TREK1 knockout mice are more sensitive than wild-type mice to pain stimulation [8]. Additionally, TREK1 knockout mice are more sensitive to mechanical stimulation than wild-type mice, making them more susceptible to tactile stimulus-induced pain. Hypersensitivity of pain receptors and temperature receptors are affected by inflammatory mediators [9]. However, under the condition of neuropathic pain, whether the expression of TREK1 channel protein in ACC neurons and the channel current are changed, and their contributions in mediating the formation of ACC neuron nociceptive sensitization remains unexplored. To clarify the role of the TREK1 channel in neuropathic pain and clarify the ion channel mechanism of ACC neurons in nociceptive sensitization, this study detected the expression and current changes of TREK1 protein in ACC neurons of CCI rats.

The function of the ACC in encoding pain information has been confirmed, and there are multiple receptors and protein molecules activated in chronic pain. TREK1 channel is widely expressed in the ACC, and changes in its expression can affect the excitability of neurons. Therefore, we proposed the following hypothesis: neuropathic pain caused by peripheral nerve injury could inhibit the expression of TREK1 in ACC neurons. Under the action of PKA, the serine at position 333 at the C end of the TREK1 channel was phosphorylated to reduce the current in the TREK1 channel, thereby enhancing the release frequency of ACC neurons and participating in the modulation process of cortical central sensitization. Combined with our existing experimental basis (pain threshold behavior means, patch clamp technique, and Western blot method), and by studying the ACC TREK1 channels electrophysiological properties of neurons and changes in protein expression in neuropathic pain, we could more deeply understand the mental derangement rational molecular mechanism of the pain of central sensitization, contributing to clarifying the role of ACC in pain regulating mechanism in the plasticity.

## 2. Materials and Methods

### 2.1. Chronic Sciatic Nerve Constrictive Injury Model (CCI)

SD rats with clean grade were randomly divided into the CCI group and the Sham group (control group). Rats in the CCI group were separated from the left sciatic nerve under combined anesthesia of ketamine and gently ligated with No. 6 silk thread to establish a neuropathic pain model in rats, while those in the Sham group were exposed only to the sciatic nerve without ligation [10]. The von Frey probe and plantar test thermal stimulation thresholds were determined 1 day before surgery and 1, 3, 5, 7, and 14 days after surgery. This study was performed in accordance with the Guide for the Care and Use of Laboratory Animals. The research protocol was reviewed and approved by the Ethical Committee of Xinhua Hospital Affiliated to Shanghai Jiaotong University School of Medicine.

### 2.2. Immunofluorescence

The rats were perfusion beheaded after depth of anesthesia, and then isopentane was used for quick-frozen at −20°C. Subsequently, the freezing microtome sections in thickness of 10 microns were prepared, and sticked on the poly lysine package. The samples were treated with 4% paraformaldehyde fixed phosphate buffer for 15 min, and 0.01 mol/L PBS 0.25% Triton-X100 broken film was added after rinsing, after which 10% bovine serum albumin (BSA) was obatained for closing for 2 h at room temperature. Then, the samples were incubated with antibodies that included TREK-1 (1:200), glial fibrillar acidic protein (GFAP, 1:200), at 4°C overnight. As a negative control of TREK1 protein, immunopeptides were used to block the specific binding of the primary antibody to the antigen. After 0.01 mol/L PBS rinse, the secondary anti-cy3-labeled goat anti-mouse antibody was added to avoid light and incubated at room temperature for 1 h. The expression of TREK1 protein was observed under Olympus BX51 fluorescence microscope, and the changes in the expression of TREK1 channel in the ACC region of neuropathic pain rats were compared.

### 2.3. Western Blot

Western blot was used to detect the changes in the expression levels of TREK1 channel protein and serine Ser333 phosphorylation in the ACC of neuropathic pain rats. SD rats were randomly divided into CCI group (16 rats) and Sham group (16 rats). Unilateral sciatic nerve was ligated by CCI group, and only sciatic nerve was exposed in Sham group without ligation. Rats were decapitated, and fresh ACC specimens were isolated and stored in liquid nitrogen. 100 mg tissue was homogenized in 1 ml phosphorylated protein lysate and centrifuged at 14000 g and 4°C for 20 min. The supernatant was the total protein and was quantified with bicinchoninic acid (BCA) protein quantitative kit. Total protein samples were collected and separated by 10% sodium dodecyl sulfate-polyacrylamide gel electrophoresis. Then, the samples were transferred to polyvinylidene fluoride (PVDF) filter membrane (Roche, Basel, Switzerland), and electrochemiluminescence (ECL) detection kit that provided sealing fluid was used for closing the membrane at 4°C overnight. The next morning, the membrane was incubated with the rabbit anti-TREK1 antibody at room temperature for 2 h, and then the corresponding secondary antibody labeled with horseradish peroxidase was incubated at room temperature for 1 h. The antibodies used in this study were anti-TREK1 antibody (Abcam, 1/1000, cat. no. ab90855) and anti-GAPDH antibody (Abcam, 1/2500, cat. no. ab9485). The membrane washing procedure was carried out according to the instructions of the kit. The immune response band was developed on the negative using ECL developer, and the image analysis software (Bio-Rad Quantity One, Hercules, CA, USA) was used for quantitative analysis.

### 2.4. Patch Clamp

The ACC was isolated under the spectromicroscope and placed in a bath containing 0°C artificial cerebrospinal fluid (ACSF) by a vibrating slicer (MA752, Campden Instruments, USA). ACSF components (mmol/L) were: 140 NaCl, 5 KCl, 20 NaHCO_3_, 1 NaH_2_PO_4_, 2 CaCl_2_, 2 MgSO4, glucose 10 mmol/L, and pH 7.4. The samples were maintained at 95% O_2_ and 5% CO_2_ mixture environment to balance for 30 min at room temperature. Then, electrode liquid (135 KCl, NaCl, 2 MgCl_2_, 5 EGTA, 10 Hepes, 0.5 EGTA, pH 7.25) was filled, and patch clamp amplifier (AxON200 B, USA) with glass microelectrode connection that contained 4–10 MΩ cutting-edge impedance was used to adjust the three-dimensional hydraulic manipulator electrode tip in contact with the cell surface. High impedance were formed by pressure suction. Composition of the external solution of the electrode (mmol/L): 140 NaCl, 5 KCl, 2 CaCl_2_, 2 MgCl_2_, 10 glucose, 10 Hepes, 25 TEA, 0.5 CdC1, PH 7.4. Except for the description, all the recording modes adopted were cell adhesion. Single-channel current is sampled online by a patch clamp amplifier supported by Digit data 1320 (AXON, USA). The channel activity was measured and analyzed with PCLAMP 11.0 program, and the sampling rate was 5–10 kHz. 5 mmol/L 4-ap was added to the electrode solution to block Ito and IKur, and 0.5 mmol/L CdCI and 25 mmol/LTEA were added to the extracellular solution to block ICa_2_+ and IK1. The clamp potential was −40 mv, and the experimental potential was −120 ∼ +80 mV, increasing at a step of 20 mV. According to the histogram of current distribution amplitude, the single-channel current amplitude value at the corresponding potential was fitted, and the i-v curve was drawn to obtain the slope conductance of the single channel.

### 2.5. Statistical Analysis

Results were performed using Statistical Product and Service Solutions (SPSS) 19.0 (SPSS Inc., Chicago, IL, USA) and presented as the mean ± SD (standard deviation) from three independent experiments. A value of *P* < 0.05 was considered to indicate a statistically significant difference.

## 3. Results

### 3.1. TREK1 Channel Expression Was Decreased in CCI Model

We investigated the effect of TREK1 expression in the ACC neurons of CCI rats, as shown in Figure 1. The immunohistochemistry analysis showed that the expression of TREK1 protein in the ACC neurons of CCI rats was 44.2 ± 0.031. However, the expression of TREK1 protein in the ACC neurons of Sham group rats was 8.3 ± 0.012. The TREK1 protein in the CCI group significantly decreased compared to that in the Sham group. These results suggested that TREK1 protein expression decreased in CCI rats.

### 3.2. The Protein Expression of TREK1 Channel Was Decreased after 7 d and 14 d of CCI Establishment by Western Blot

Then, the expression of TREK1 in different time points after induction of CCI was detected. It was observed that the expression of TREK1 channel was increased after 1 d of model establishment, where asits expression was remarkably decreased in the ACC neurons of CCI rats after 7 d and 14 d (Figure 2).

### 3.3. The TREK1 Channel Current Was Decreased in ACC Cortical Neuron

After the patch clamp was completed to detect the changes in the current of the TREK1 channel of neurons in the ACC region of CCI rats, the TREK1 channel was decreased by local administration of drugs in the ACC of CCI rats (Figure 3).

### 3.4. Local Administration of LIN Reversed Pain Threshold Behavior of CCI Rats and Expression of TREK1 Channel Protein in ACC

As shown in Figure 4, we investigated the changes in pain threshold behavior and expression level of TREK1 between two groups. The TREK1 channel was activated by local administration of LIN in ACC of rats, and changes in pain threshold of CCI rats were detected. Western blot analysis results suggested that the TREK1 channel protein expression level was significantly downregulated in the ACC region after administration. The changes of the phosphorylation level of TREK1 channel serine in ACC of CCI rats after local administration of LIN were measured by Western blot.

## 4. Discussion

Functional imaging and electrophysiological studies have shown that ACC neurons are activated when nociceptive stimulation or hypnotic suggestion is given to test volunteers to simulate nociceptive stimulation [11, 12]. However, inhibition of the excitatory synaptic transmission of ACC neurons can significantly reduce the responsiveness of pain-related emotions and have analgesic effects. The analysis of extracorporeal brain slice showed that the excitability of ACC neurons can be sustained for a long time in chronic pain. Long-duration facilitation can be induced in the local stimulation of ACC in amputated rats, while the expression of NMDA receptor subunit NR2B in the ACC of inflammatory pain rats is activated [13]. In neuropathic pain models caused by peripheral nerve injury, the firing frequency of intermediate neurons in ACC brain slices changes, but other electrophysiological characteristics of neurons are not affected [5]. Using patch clamp in vivo, nociceptive stimulation could change the firing of ACC pyramidal neurons but had no response to non-nociceptive stimulation [14]. We used intracellular electrophysiological records to clarify the changes of ACC neuron membrane in nociceptive stimulation. However, the ion channel mechanism affecting the electrophysiological characteristics of ACC neurons has not been further studied.

Potassium channels are necessary for triggering action potentials and play an important role in the release of synaptic transmitters [15]. Current studies have shown that voltage-sensitive, calcium-sensitive, and sensitive potassium channels are closely related to the occurrence of neuropathic pain and are involved in the formation of central sensitization [16, 17]. In recent years, the study reported a new class of potassium channels.Unlike traditional potassium ion channel, it has four cross diaphragm and two channel structure domain, therefore is called double orifice potassium channels (two-pore-domain potassium channels, K2P).Studies have confirmed that the double hole in the family of potassium channels TREK1 channel is widely expressed in rat cerebral cortex and spinal cord dorsal horn neurons, which could adjust the excitability of the neurons and the neurotransmitter release.Moreover, these features may be associated with the pathogenesis of chronic pain [7, 18]. TREK1 channel could be regulated by pain stimulation, including pressure and heat. TREKl knockout mice are more sensitive to pain stimulation than wild-type mice. The dorsal root ganglion neurons increased sensitivity to thermal stimulation, and giving cold stimulus exhibited no effects on TREK1 channels expression, suggesting that TREK1 may not participate in the cold feeling [19]. This study detected the expression and current changes of TREK1 channel protein in ACC neurons of CCI rats to clarify the role of TREK1 channel in neuropathic pain and clarify the ion channel mechanism of ACC neurons in nociceptive sensitization.

TREK1 channel is related to resting potential and is involved in regulating the overall excitability of neurons, which is easily affected by mechanical stimulation, acid-base balance, body temperature, and other factors. Protein kinase A (PKA) phosphorylates Ser333 at TREK1C end through the second messenger cAMP, causing the closure of TREK1 channel. Protein kinase C (PKC) can also phosphorylate Ser333 and Ser300 residues at the C end of the TREK1 channel, thus shutting down the TREK1 channel [7, 20]. TREK1 channel may be involved in the occurrence and development of ACC neuron nociceptive sensitization through the following two ways: the depolarization of presynaptic neurons can activate the voltage-dependent calcium channel and increase the calcium influx, and depolarization of postsynaptic neurons can reduce the blocking effect of Mg on NMDA receptors, thus increasing the excitability of neurons [21]. Peripheral nerve injury enhances synaptic transmission and increases intracellular cAMP level, and serine at position 333 of TREK1 channel C is phosphorylated by protein kinase A, leading to the closure of the channel, which impedes the outflow of potassium ions and increases the excitability of neurons [7].

In the present study, neuropathic pain caused by peripheral nerve injury could inhibit the expression of TREK1 channel in ACC neurons. Under the action of PKA, the serine at position 333 at the C end of the TREK1 channel is phosphorylated to reduce the current in the TREK1 channel, thereby enhancing the release frequency of ACC neurons and participating in the modulation process of cortical central sensitization. Combined with our existing experimental basis (pain threshold behavior means, patch clamp technique, and Western blot method), this study focuses on the ACC TREK1 channels electrophysiological properties of neurons and changes in protein expression in neuropathic pain, aiming at comprehensively understanding the mental derangement rational molecular mechanism of pain of central sensitization, and elucidating the role of ACC in pain regulating mechanism in the plasticity is of great significance.

The study also has some limits. What regulates TERK1 is not clear, and further in vitro study is also needed to provide deeper insights.

## 5. Conclusion

In summary, the expression of TREK1 channel protein was inhibited in neurons in the ACC area of the CCI cortex of rats and the current of TREK1 channel was decreased, which played an important role in the regulation of neuropathic pain.

## Figures and Tables

**Figure 1:** The percentage of TREK1-positive cells was detected by immunofluorescence. The values were accordance with normal distribution, so Student's t-test was used to compare the differences between the Sham group and CCI group (n=12).

**Figure 2:** The change of TREK1 expression in the ACC neurons was detected by Western blot at 1, 3, 7, and 14 days (n=12).

**Figure 3:** The changes of TREK1 channel current in ACC cortical neuron. The current of the TREK1 channel of neurons between two rats was detected by patch clamp, and the results showed that the TREK1 channel between two groups was significantly activated by local administration of drugs (*n* = 6).

**Figure 4:** The changes in pain threshold behavior of CCI rats and expression of TREK1 channel protein in ACC. The TREK1 channel was activated by LIN. Paw withdraw threshold value and Paw withdraw latency for Sham, CCI, and LIN groups after 1, 3, 5, 7, 14, and 21 days were detected. Treld positive rate, GFAP positive rate, NEUM positive rate, and current for three groups of rats were detected. The level of TERK1 protein in the ACC neurons was assessed by Western blot at 1, 3, 7, and 14 days.

## Data Availability

The datasets used and analyzed during the current study are available from the corresponding author on reasonable request.
